# Acupuncture regulates the glucose metabolism in cerebral functional regions in chronic stage ischemic stroke patients---a PET-CT cerebral functional imaging study

**DOI:** 10.1186/1471-2202-13-75

**Published:** 2012-06-27

**Authors:** Yong Huang, Chunzhi Tang, Shuxia Wang, Yangjia Lu, Wei Shen, Junjun Yang, Junqi Chen, Renyong Lin, Shaoyang Cui, Huiling Xiao, Shanshan Qu, Xinsheng Lai, Baoci Shan

**Affiliations:** 1 School of Traditional Chinese Medicine, Southern Medical University, Guangzhou, China; 2 Department of Acupuncture and Massage, Guangzhou University of Traditional Chinese Medicine, Guangzhou, China; 3 Department of Nuclear Medicine, Canton Provincial People’s Hospital, Guangzhou, China; 4 Department of Acupuncture and Rehabilitation, Guangdong Provincial Second TCM Hospital, Guangzhou, China; 5 Key Laboratory of Nuclear Analytical Techniques, Institute of High Energy Physics, Chinese Academy of Sciences, Beijing, China

**Keywords:** Waiguan (TE5), Sham point, Ischemic stroke, Needling/sham needling, PET-CT cerebral functional imaging, Cerebral activating/deactivating effect

## Abstract

**Background:**

Acupuncture has been applied to aid in the recovery of post-stroke patients, but its mechanism is unclear. This study aims to analyze the relationship between acupuncture and glucose metabolism in cerebral functional regions in post-stroke patients using ^18^ FDG PET-CT techniques. Forty-three ischemic stroke patients were randomly divided into 5 groups: the Waiguan (TE5) needling group, the TE5 sham needling group, the sham point needling group, the sham point sham needling group and the non-needling group. Cerebral functional images of all patients were then acquired using PET-CT scans and processed by SPM2 software.

**Results:**

Compared with the non-needling group, sham needling at TE5 and needling/sham needling at the sham point did not activate cerebral areas. However, needling at TE5 resulted in the activation of Brodmann Area (BA) 30. Needling/sham needling at TE5 and needling at the sham point did not deactivate any cerebral areas, whereas sham needling at the sham point led to deactivation in BA6. Compared with sham needling at TE5, needling at TE5 activated BA13, 19 and 47 and did not deactivate any areas. Compared with needling at the sham point, needling at TE5 had no associated activation but a deactivating effect on BA9.

**Conclusion:**

Needling at TE5 had a regulating effect on cerebral functional areas shown by PET-CT, and this may relate to its impact on the recovery of post-stroke patients.

## Background

Acupuncture is an important part of traditional Chinese medicine and has been used for the treatment and recovery of stroke patients. Recently, it has been proven to have a positive effect on post-stroke patients in multi-center studies involving large datasets of clinical observations and evidence-based literature analyses [1-6]. However, the underlying mechanism of this relationship is still unclear.

There are numerous methods to study the mechanisms of treating stroke by acupuncture. We focused on cerebral functional imaging because it enables observation of the real-time effects of acupoint needling and the reactions of functional brain regions in humans instead of in the animal brain.

Cerebral functional imaging has been successfully combined with acupuncture researches. Needling at acupoints can activate particular cerebral areas under physiological conditions in both humans and monkeys [7-14]. Needling can also result in activation patterns that closely relate to areas involved with the treatment of depression, vascular dementia, rheumatoid arthritis, functional dyspepsia and Parkinson’s disease [9,10,15-18]. In addition, the response of the brain to needling at a single acupoint and needling at acupoints in different meridians or different regions has been studied [19-26] and compared with true, sham and different manipulations of needling [27-30].

Studies based on cerebral functional imaging during acupuncture needling of stroke patients have been published previously. Acupuncture-related activation changes in certain cerebral functional areas of stroke patients have been observed. He et al. reported activations in the primary motor area, premotor area, primary sensory area, superior parietal lobe, superior temporal gyrus and insula of the opposite hemisphere as well as bilateral activation of the sensory areas and the affected areas when patients were asked to move their index finger while being needled at Quchi (LI11) and Shousanli (LI10) on the side affected by hemiparalysis [31]. The study of He et al. did not involve any control factors and was only an observation of needling.

The effect of the special acupuncture therapies commonly used to treat chronic stage stroke patients also has been studied. Wang F, et al. observed a significant difference in the effect of needle retention and electro-acupuncture stimulation on the contralateral cerebral hemisphere cortex and thalamus, ipsilateral basal ganglion and bilateral cerebella: specifically, the change in cerebral blood flow induced by electro-acupuncture was greater than that induced by needle retention [14]. Schockert T, et al. published that Yamamoto new scalp acupuncture could affect certain cortical activations [32]. Zhang et al. compared Xingnao Kaiqiao acupuncture with routine needling and found that the former had a stronger effect on the activation of cerebral functional regions [26]. Special therapies of acupuncture are worthy topics of study, but studies should ideally begin with the fundamental relationships between needling at one acupoint and the changes in brain functional areas.

The different effects of true and sham needling were investigated. Li et al. reported that both electro-acupuncture and the touch of the needle tip on the skin in stroke patients and healthy volunteers resulted in the activation of the primary and secondary sensory centers, the motor center and cerebellum [33]. However, the effects of needling stroke patients as well as the needle-tip-touching stimulation resulted in the strongest signals [33]. Jeun SS, et al. observed that needling at GB34 could stimulate bilateral sensorimotor areas (BA 3, 4, 6 and 7), whereas very few areas were activated when sham stimulation was given [11]. Schaechter et al. found a significant positive correlation between changes in the function of the affected upper limb (spasticity and range of motion) and activation within a region of the ipsilesional motor cortex in patients treated with acupuncture relative to patients treated with sham acupuncture [34]. The use of sham needling as the control factor strengthens the study, but it is not enough; needling on a sham point should also be included.

The effect of treating post-stroke aphasia patients with acupuncture and the relationship between acupuncture and cerebral functional regions were studied. Li et al. and Chau et al. observed that language-deficit-implicated acupoint stimulation could selectively activate the brain on the lesion side in post-stroke aphasia patients [35,36]. These studies highlighted the use of acupuncture in the study of post-stroke patients.

The above researches suggest that acupuncture can be applied to treat chronic stroke patients, and hence, in this study, we selected post-ischemic patients with the ischemic lesions limited to the left internal capsule, and the symptoms manifested as abnormal movements and sensations of the right limbs.

The published paper focused on some acupoints that are good for the recovery of stroke patients, including Waiguan (TE5) [11,14,26,31-34]. TE5, can aid in the patient’s recovery of movement, sensation and speaking and treat dysfunctions of the eyes, ears and mental activities. In this study, we targeted TE5 on the right side of the patient and tried to analyze its action on regional cerebral functional areas.

The published studies described above have utilized PET, SPECT and fMRI but not PET-CT. We used PET-CT as the examination method because it provides high spatial discrimination.

Our observations included pure needling and a comparison between needling and sham needling, which provided stronger evidence for the underlying mechanisms. In this experiment, we included a sham needle as well as a sham point, to clarify the distinction between the action of acupuncture and the selected acupoint.

The former studies focused on specialized acupuncture techniques or special groups of acupoints. In this experiment, only one acupoint, TE5, and only one technique, twisting, were involved to simplify the experimental condition and illustrate the mechanism more easily.

Previous research has focused on post-stroke patients with aphasia and found that acupuncture could affect the language-related cerebral regions. The current experiment involves patients with left hemisphere ischemic damage accompanied by light aphasia in addition to typical hemiplagia. The acupoint TE5 can potentially help the recovery of language as well as address the abnormal motion and sensation of affected limbs.

Thus, in this study, we execute needling at a single acupoint and compare the results with sham needling and needling at a sham point. In this way, we tried to find the “special activated/deactivated cerebral functional regions” resulted from needling, target cerebral functional regions needling at TE5 acting on, and then related these changed cerebral areas to the cerebral areas that involved in the recovery of stroke patients, in order to explain the mechanism of needling to help the recovery of hemiplegia.

The acupoint used in the experiment was TE5, a commonly used one in the treatment of stroke patients. Only one acupoint was adopted in this study, even if a group of acupoints were usually applied in the clinical practice of stroke treatment. The basic mechanism study should be begin with a single point, and develop as “single point—two points grouping—more points grouping”. In the mean time, it was convenient for us to process the “block stimulation” strictly.

## Results

All 45 patients finished the PET-CT scan under different states. Among them, a patient from Group 3 who received needling at the sham point and another patient from Group 4 who received sham needling at the sham point did not remain immobile during the scan, and the images were blurred due to large movements of the patient’s head. The datasets were removed from the study, and the remaining 43 patients’ data were processed.

### Comparison between true and non-needling at TE5

Compared with non-needling, needling at TE5 resulted in activation of BA30, whereas sham needling at TE5 and needling/sham needling at the sham point did not lead to any cerebral activation. Needling/sham needling at TE5 and needling at the sham point did not deactivate any cerebral areas, but sham needling at the sham point led to a deactivation of BA6 (Table 1 and Figures 1 and 2).

**Table 1:** Actived/deactivated cerebral areas by needling vs. non-needling

**Stimulating style**	**Brain areas**	**BA**	**Activated/deactivated**	**Talairach (mm)**			**T**
				**X**	**Y**	**Z**	
Needling at TE5	Left cerebrum, Limbic Lobe, Posterior Cingulate	30	activated	−4	−62	12	4.09
Sham needle at sham point	Right Cerebrum, Frontal Lobe,Middle Frontal Gyrus	6	deactivated	30	10	60	5.50

**Figure 1:** Cerebral areas activated by needling at TE5 vs. non-needling (red areas).

**Figure 2:** Cerebral areas activated by sham needling at the sham point vs. non-needling (red areas).

### Comparison between true and sham needling at TE5

Compared with sham needling at TE5, needling at TE5 activated BA13, 19 and 47 and did not deactivate any areas (Table 2 and Figure 3).

**Table 2:** Cerebral areas activated by needling vs. sham needling at TE5

**Brain areas**	**BA**	**Talairach(mm)**			**T**
		**X**	**Y**	**Z**	
Right Cerebrum, Occipital Lobe, Middle Temporal Gyrus	19	36	−58	14	6.43
Right Cerebrum, Frontal Lobe, Inferior Frontal Gyrus	47	62	20	−4	4.88
Right Cerebrum, Frontal Lobe, Inferior Frontal Gyrus	47	58	24	−10	4.34
Right Cerebrum, Sub-lobar, Insula	13	30	−26	22	4.64
Right Cerebrum, Sub-lobar, Insula	13	34	−34	24	4.29

**Figure 3:** Cerebral areas activated by needling vs. sham needling at TE5 (red areas).

### Comparison between needling at TE5 and at the sham point

Compared with needling at the sham point, needling at TE5 did not have any activating effect, but it did have a deactivating effect on BA9 (Table 3 and Figure 4).

**Table 3:** The cerebral areas deactivated by needling at TE5 vs. needling at the sham point

**Brain areas**	**BA**	**Talairach(mm)**			**T**
		**X**	**Y**	**Z**	
Left Cerebrum, Frontal Lobe, Medial Frontal Gyrus	9	−14	38	28	4.65
Right Cerebellum, vermis		18	−64	55	4.42

**Figure 4:** Cerebral areas deactivated by needling at TE5 vs. at the sham point (red areas).

## Discussion

As mentioned above, it is popular to treat chronic stage ischemic stroke patients with acupuncture in China [1-6]. One of the commonly targeted acupoints for the treatment is TE5. According to the theory of meridians and acupoints, acupuncture at TE5 has been shown to have curative effects on limbic paralysis and pain, dysfunction of the eye and ear, migraine, costal pain, fever and mental disorders, which indicates that it not only helps hemiplegia patients with motor recovery, but it also may ameliorate sensory dysfunction, post-stroke depression, dementia, aphasia, visual dysfunction, auditory dysfunction and sleeping disorders ([37,38]).

Patients involved in this experiment received needling at TE5. To prove the relationship between needling at TE5 and the activation/deactivation of cerebral functional regions, patients without any needling, with needling at a sham point and with sham needling at TE5 were included as control groups.

The study showed that, compared with non-needling, sham needling at TE5 and needling or sham needling at the sham point did not have any effect on the functional regions of the brain. In contrast, needling at TE5 resulted in activation of BA30, a part of the limbic system, which indicates that needling at TE5 in ischemic stroke patients could specifically act on the limbic system.

Compared with non-needling, needling and sham needling at TE5 and needling at the sham point did not have any deactivating effects on the brain. One exception to this was observed in BA6, which was deactivated when sham needling was done at the sham point. BA6 is a motor center and takes part in the planning and execution of motor function. According to clinical experience, needling at TE5 can produce the strongest curative effect, followed by sham needling at TE5, then needling at the sham point, while sham needling at the sham point generally has the smallest effect. Our experiment proved that sham needling at the sham point, which produced the lightest curative effect, led to the deactivation of BA6 in ischemic stroke patients.

Sham needling has been used as a control in some acupoint needling studies [39]. The way it is implemented or manipulated can vary, and it is not a standard part of every study [40,41].

Compared to sham needling at TE5, needling at TE5 was shown to activate BA13, 19 and 47, but it did not lead to any deactivation, which indicates that there is a difference between true and sham needling. BA13, 19 and 47 are located in the right hemisphere and participate in cortical association, vision processing and motor execution, respectively. Unlike sham needling, true needling acts specifically on functional areas related to vision and motor execution of the right hemisphere, the healthy side of the brain, and this may be related to the mechanism underlying the role of acupuncture in the recovery from left internal capsule ischemia.

There are different reports on the comparison between true and sham needling. Recently, a systematic review indicated that acupuncture may be no more effective than sham acupuncture in treating temporomandi-bular joint disorders [42]. But a study on post-hemorrhoidopexy showed, acupuncture was better that both sham acupuncture and conventional analgesia group (Langenbach et al., [43]). A fMRI study found that acupuncture at Sanyinjiao (SP 6) was different from needling at the sham point based on the analysis of resting-state amplitude of low-frequency fluctuation in sleep deprivation volunteers (Dai et al,. [44]). According to TCM theory, sham needling also stimulated the “cutaneous region” of meridians (the Qi of the meridian distributes to the skin centered on the meridian and diffuses to other nearby meridians), similar to transcutaneous stimulation, which may lead to a certain curative effect.

Our group also made a comparison between true and sham needling at TE5 in volunteers, and found the different activated areas were left BA13 and 42 and the cerebellum by the PET scan (Lai X et al,. [29]). We found that acupoint needling effects manifested differently under the healthy or pathological conditions. Compared to sham needling, true needling at TE5 in stroke patients mainly affect the healthy hemisphere and in this way to help the recovery of stroke.

Compared to needling at the sham point, needling at TE5 did not lead to activation, but it did lead to deactivation of BA9 and the right cerebellum. BA9, located in the both hemispheres, is involved in govern execution. This experiment shows that needling at TE5 is different from needling at the sham point. Needling at TE5 caused deactivation of the cognitive execution center of the left brain (the diseased side) and deactivation of the right cerebellum, which is related to the planning and execution activity on the healthy side.

Sham point, also called as non-acupoint, is regarded with no curative effect even if it may have a certain (limited) curative effect because there is still some Qi distributed to the border of the two meridians’ basins. Now it is used as a control involved in the acupucnture research. Recent studies showed the difference between needling at a true acupoint and a sham point. Stimulation at true acupoints elicited a greater response than that of non-acupoints in cardiovascular disease (Tjen-A-Looi et al,. [45]). Also the differences were found in the actions on the cerebral functional areas proved by brain imaging ([46]; Napadow et al,.2009).

The sham point used in this study was located between two meridians but did not belong to any meridians. The comparison showed that the difference between needling at the true and sham points concentrated to cognition of planning and execution activities. TE5 has the function of treating mental disorders ([37,38]), which was manifested in this experiment in the treatment of post stroke patients, compared with the sham point needling.

We have observed the specific action of needling at TE5 on cerebral functional regions of ischemic stroke patients compared to non-needling, sham needling at TE5 and needling at the sham point (Table 4).

**Table 4:** Summary of the cerebral areas activated/deactivated by needling at TE5

**Left brain (affected hemisphere)**	**Right brain (healthy hemisphere)**
*Frontal Lobe, Medial Frontal Gyrus*	Frontal Lobe,Inferior Frontal Gyrus
Limbic Lobe,Posterior Cingulate	Occipital Lobe, Middle Temporal Gyrus
	Sub-lobar,Insula
	*Cerebellum*

Note: italics = deactivated areas.

Our results indicate that needling at TE5 activates brain areas that are involved in motor execution, vision and emotion and that are predominantly located in the healthy hemisphere. There is also a trend indicating that needling of TE5 on the right side in patients with left hemisphere ischemia could activate the areas of motor execution in the healthy hemisphere while simultaneously deactivating areas related to motor execution in the affected hemisphere. In addition, needling at TE5 led to the deactivation of the cerebellum on the healthy side and BA9 of the affected side of the brain.

Deactivation, compared to the condition of baseline, the glucose metabolism is negative, which indicates a re-distribution of the attention resource (Seo J et al., [47]). BA 9 has close relationship with an organization of an execution. Cerebellum controls the movement, sensation and cognition (Habas C et al., [48]). Compared to needling at the sham point, needling at the true acupoint could reduce the glucose metabolism of the cerebral area which controls the execution of affected hemisphere, in the mean time reduce the glucose metabolism of cerebellum of the healthy hemisphere. It was inferred that needling at TE5 resulting a re-distribution of glucose in order to help the recovery of stroke.

The results indicated that needling at TE5 had a regulating action to the glucose metabolism of cerebral functional areas. In order to help the recovery of stroke patients, needling at TE5 increased the glucose metabolism of the healthy hemisphere and decrease it of the affected side, which meant that needling at TE5 had a general regulation to the brain without focused on the affected local area.

## Conclusion

We have attempted to explain the mechanism of treating chronic stage ischemic stroke patients with needling at TE5 with observations relating needling at TE5 with specific brain activations and deactivations. We found that needling at TE5 in stroke patients could activate motor execution- and vision-related cerebral regions in the healthy hemisphere and the limbic system of the affected hemisphere and also deactivate the motor execution-related cerebral region of the affected hemisphere and the cerebellum of the healthy hemisphere. Needling at TE5 could improve the glucose metabolism of the healthy hemisphere while decreasing the glucose metabolism of the affected hemisphere, and this may be the mechanism underlying the role of acupuncture in the recovery of hemiplegia.

## Methods

### Clinical data

Forty-five ischemic stroke patients from the first and second affiliated hospitals of Guangzhou Traditional Chinese Medicine (TCM) University, Yuexiu District Peoples’ Hospital and Canton Provincial Peoples’ Hospital, were diagnosed using ICD-9 434 and ICD-8 433 [49]. Their National Institutes of Health Stroke Scale (NIHSS) scores were 7–15 [50].

The inclusion criteria were as follows: (1) the patient was suffering from ischemia in the left internal capsule, as shown by CT or MR imaging, that manifested as typical hemiplegia of the right side; (2) the patient had passed the acute stage and was in the sequela stage with NIHSS scores of 7–15 [50]; (3) the patient was aged between 40 and 65 years; (4) the patient was taking aspirin enteric-coated tablets 100 mg/d and famotidine 20 mg/d as a basic treatment and controlled their blood pressure, cholesterol and sugar; (5) the patient ate and slept regularly, did not smoke excessively or drink tea or coffee excessively and had a body mass index within 18.5-22.9 [51]; (6) the patient was right-handed; and (7) the patient had given informed consent after being informed of the study protocol, which was approved by the Ethics Committee of the first affiliated Hospital, Guangzhou University of TCM, and registered on the website of the Chinese Clinical Trial Registry (ChiCTR- NRC- 00000255).

The exclusion criteria were as follows: (1) serious diseases, such as dysfunction of the heart, liver or kidney, serious infection, malignant hypertension or malignant tumor; (2) serious aphasia, unconsciousness or mental disorders (including fear of confined spaces), which could affect their cooperation during the experiment; (3) painful diseases (including dysmenorrhea) or the use of analgesic medicines that could affect brain metabolism; (4) (for women) pregnancy or lactation; (5) weakness that prevented the patient from completing 4 hours of fasting; (6) diabetes, with the possible need for anti-diabetic drugs during the 4 hours prior to the PET-CT scan, or the inability to control blood sugar at levels under 8.3 mmol/L (150 mg/dL); (7) thrombocytopenia or hemophilia, which are both counterindications for acupuncture; and (8) non-sensitivity or over-sensitivity to needling versus sham needling sensations as determined at a screening test 3 months prior to the study.

The patients in the study included 26 males and 19 females, with an average age of 56.10士3.41 years, average NIHSS score of 10.82士2.32, and average disease history of 3.20士1.20 years.

### Experiment methods

#### Needling methods

The patients were randomly divided into 5 equal groups of 9 subjects each: the needling TE5 group, the sham needling TE5 group (9 cases), the needling sham point group (9 cases), the sham needling sham point group (9 cases) and the non-needling group (9 cases) (Table 5). Both true and sham needling were performed by the same physician who conducted the patient screening 3 months prior to the start of the study.

**Table 5:** Ischemic stroke patient groups (x ± SE)

**Groups**	**N**	**Age (year)**	**Sex (F/M)**	**Disease history (month)**	**NIHSS**
Group 1					
Needling TE5	9	55.78 ± 3.90	5/4	3.45 ± 1.00	10.30 ± 3.72
Group 2					
Sham needling TE5	9	56.34 ± 4.18	5/4	3.12 ± 2.21	11.89 ± 3.56
Group 3					
Needling sham point	9	56.54 ± 4.15	5/4	3.32 ± 1.66	10.42 ± 2.15
Group 4					
Sham needling sham point	9	57.67 ± 4.36	6/3	2.95 ± 1.13	9.50 ± 3.10
Group 5					
Non-needling	9	54.17 ± 4.66	5/4	3.16 ± 1.10	11.95 ± 2.33

TE5 on the patient’s right side was located as described in the Name and Location of Acupoints: Chinese National Standard (General Administration of Quality Supervision, [52]). The location of TE5 was identified as 2 cun (cun is a special length unit in acupuncture referring to the width of the interphalangeal joint of the patient’s thumb) above the transverse crease of the dorsum of the wrist between the radius and the ulna on the forearm. The sham point was located on the middle point of the horizontal line crossing TE5 and the Small Intestine Meridian of Hand-Taiyang on the patient’s right side (Figure 5). 

**Figure 5:** Location of TE5 and the sham point.

True needling: the skin around the TE5 or sham point was sterilized, and a needle was inserted by the physician using the tube insertion method (the needles and tubes were acquired from DONGBANG AcuPrime Co., UK). The auxiliary part of the tube was placed on the skin, and the needle was placed into the matching tube over the acupoint/sham point; then, the end of the needle was tapped to make the tip of the needle go through the skin. The tube was then removed, and the needle was punctured to a depth of 15 ± 2 mm; the handle was then twisted to produce the needling sensation. The physician then manually stimulated the needle with an even force, and reduced manipulation was applied by twirling the needling 180° 60 times/min over 3 min. The needle position was then maintained in the absence of twirling for 5 min. The procedure was repeated 3 times for a total of 24 min.

Sham needling: the procedures for sterilization of TE5 or the sham point and the application of needling instruments were the same as described above, except that sham needles were used. The auxiliary part of the tube was applied to the skin, with a sham needle placed in the tube over the acupoint/sham point. The sham needle was then tapped to make its tip touch the skin without puncturing it. The tip of the sham needle was allowed to touch the skin for 3 min, and the needle was then lifted for 5 min. This procedure was repeated 3 times for a total stimulation time of 24 min.

Non-needling: sterilization of the local skin of TE5 and the application of the needling instruments were performed the same way as described above. The auxiliary part of the tube was applied to the skin with the tube placed directly over the acupoint but without a true or sham needle. The end of the tube was tapped with the same force as that used for a true or sham needle, and the tube was then removed.

#### PET-CT scan

A PET-CT scanner was used to collect images of the brain (Siemens Sensation Biograph Somatom 16 PET/CT, Germany). The CTIRDSIII accelerator was made by the Wei-Lun PET Diagnosis Centre of the Canton Provincial People’s Hospital. The tracer used was ^18^fluoride-deoxygluocse (^18^ F-FDG, radio-chemical purity >95%).

Injection of the tracer: intake of food in the 4 hours prior to the PET-CT examination was prohibited. Each patient wore blinders over their eyes (Xinhua Tourism Co., China) and used earplugs to block out sound (Aearo Co., USA). After the measurements of body weight, height and blood sugar, the patients were instructed to lie on a bed and rest in a quiet and dimly lit room with the temperature held between 20 to 24 °C. The tracer ^18^ F-FDG (0.14 mCi/kg) was given intravenously (bolus) 1.5 min after the needle/sham needle insertion. The needling/sham needling stimulation was done before injection. The patient was then told to rest.

The PET-CT scan was started 40 min after the injection of radioactive material. The patient’s head was placed into a supporting device, localized by a laser and fixed in a position where the superior and inferior lines were parallel to the orbitomastoid (OM) line and enclosed the cerebrum and the cerebellum.

Image collection: cerebral images were first collected by CT, with settings as follows: 120 KV, 320 mAs, pitch = 1.25, collimation = 0.75 mm, and layer thickness of the reconstructed image = 5.0 mm with a 5.0-mm spacing. PET was then performed with a 3D model, and reconstructed with the iteration method after CT attenuation correction, which resulted in the final brain images. The PET-CT scan lasted for 20 min.

The whole course was arranged as the following (Figure 6).

**Figure 6:** The processing course.

#### Data processing

The data were processed with MRIcro, Statistical Parametric Mapping software (SPM2, http://www.fil.ion.ac.uk) and the corresponding operating platform of Matlab 6.5. The images were first changed from DICOM formatting for analysis with MRIcro, and then the data were pre-processed using SPM2. The images were then normalized to the Montreal Neurological Institute (MNI) space and smoothed spatially by a Gaussian kernel of 12 × 12 × 12 mm^3^. The model was then built by analyzing the smoothed data with the generalized linear mode voxel by voxel. The corresponding *t* values for each voxel were assessed using a dual-sample *t*-test, and statistical parametric mapping was based on these *t* values (P < 0.001, uncorrected, K > 30). The changes of different cerebral regions under different stimulations were obtained and superimposed onto each patient’s standard anatomic images. Cerebral areas activated or deactivated by true or sham needling at TE5 vs. non-needling or sham needling at TE5, and that of true or sham needling at a sham point vs. non-needling were compared. The results were reported in Talairach space coordinates and activated/deactivated Brodmann (BA) areas.

## Authors’ contributions

Xinsheng Lai, Yong Huang and Chunzhi Tang planed the experiment. Yong Huang, Chunzhi Tang and Junjun Yang managed the clinical experiment. Shuxia Wang took the charge of PET-CT scan. Shaoyang Cui and Wei Shen made the clinical assessment of the involved patients. Yangjia Lu needled all the patients during the experiment. Baoci Shan worked as the head of data processing group and made the direction to the images processing. Shanshan Qu and Renyong Lin joined in the processing group, worked as the assistants. Junqi Chen and Huiling Xiao took the charge of statistics. Yong Huang drafted the manuscript. All authors read and approved the final manuscript.
